# Identification of Hub Genes to Regulate Breast Cancer Spinal Metastases by Bioinformatics Analyses

**DOI:** 10.1155/2021/5548918

**Published:** 2021-05-12

**Authors:** Yongxiong He, Yongfei Cao, Xiaolei Wang, Wu Jisiguleng, Mingkai Tao, Jianfeng Liu, Fei Wang, Lemeng Chao, Wenjun Wang, Pengfei Li, Haiping Fu, Wei Xing, Zhibo Zhu, Yanqiang Huan, Hongwei Yuan

**Affiliations:** ^1^Department of Spine Surgery, Inner Mongolia People's Hospital, Hohhot, 010017 Inner Mongolia, China; ^2^Trauma Orthopedic Department, Guizhou Provincial Orthopedics Hospital, No. 123 Shangchong South Road, Nanming District, Guiyang City, Guizhou Province, China; ^3^Department of Pathology, Inner Mongolia People's Hospital, Hohhot, 010017 Inner Mongolia, China

## Abstract

Breast cancer (BC) had been one of the deadliest types of cancers in women worldwide. More than 65% of advanced-stage BC patients were identified to have bone metastasis. However, the molecular mechanisms involved in the BC spinal metastases remained largely unclear. This study screened dysregulated genes in the progression of BC spinal metastases by analyzing GSE22358. Moreover, we constructed PPI networks to identify key regulators in this progression. Bioinformatics analysis showed that these key regulators were involved in regulating the metabolic process, cell proliferation, Toll-like receptor and RIG-I-like receptor signaling, and mRNA surveillance. Furthermore, our analysis revealed that key regulators, including C1QB, CEP55, HIST1H2BO, IFI6, KIAA0101, PBK, SPAG5, SPP1, DCN, FZD7, KRT5, and TGFBR3, were correlated to the OS time in BC patients. In addition, we analyzed TCGA database to further confirm the expression levels of these hub genes in breast cancer. Our results showed that these regulators were significantly differentially expressed in breast cancer, which were consistent with GSE22358 dataset analysis. Furthermore, our analysis demonstrated that CEP55 was remarkably upregulated in the advanced stage of breast cancer compared to the stage I breast cancer sample and was significantly upregulated in triple-negative breast cancers (TNBC) compared to other types of breast cancers, including luminal and HER2-positive cancers, demonstrating CEP55 may have a regulatory role in TNBC. Finally, our results showed that CEP55 was the most highly expressed in Basal-like 1 TNBC and Basal-like 2 TNBC samples but the most lowly expressed in mesenchymal stem-like TNBC samples. Although more studies are still needed to understand the functions of key regulators in BC, this study provides useful information to understand the mechanisms underlying BC spinal metastases.

## 1. Introduction

Breast cancer (BC) had been one of the deadliest types of tumors in women worldwide [1]. Almost 2.5 million patients were diagnosed with BC in 2018 [1]. Distant metastasis is the main cause of BC-related death, which happened in about 20% to 30% of BC patients [2]. Even though a series of novel therapies were developed for BC, the median overall survival for metastasis BC remained as short as about 40 months [3]. Thus, understanding the pathogenic mechanism of BC is still urgent to identify novel biomarkers for the prognosis and treatment.

Previous studies showed that more than 65% of advanced-stage BC patients were identified to have bone metastasis [4]. Sandor et al. found that nearly 70% of bone metastasis occurred in the spine [5]. BC spinal metastases lead to severe pain, paraplegia, and bladder and/or bowel dysfunction. BC spinal metastases seriously impair the survival, mobility, and quality of life [6]. Emerging efforts were paid to identify regulators involving BC metastasis. For instance, Bonapace et al. found that suppression of CCL2 significantly suppressed BC metastasis through the regulation of angiogenesis [7]. LIFR was identified as a BC metastasis suppressor through Hippo signaling [8]. A recent study revealed that ULK1 phosphorylates Exo70 to suppress breast cancer metastasis [9]. However, the molecular mechanisms involved in the BC spinal metastases remained largely unclear.

Recently, microarray showed significant advances in the understanding of pathological causes of human cancers. A few studies have identified BC-related genes using public datasets. For example, Tang et al. identified key genes involved in BC brain metastasis using GSE100534 and GSE52604 [10]. Zeng et al. identified key pathways in response to trastuzumab treatment in BC using GSE22358 [11]. Here, we conducted an analysis of the GSE26338 dataset to identify BC spinal metastasis-related key genes. This study could provide novel information to identify biomarkers for the prognosis and treatment of BC.

## 2. Material and Methods

### 2.1. Microarray Data

The microarray gene expression dataset GSE26338 [12] was obtained from the GEO database. Principal component analysis (PCA) was conducted to evaluate similarity among normal, BC, and BC spinal metastasis samples. The clinical data of breast cancer patients were obtained from previous studies [12, 13]. The limma R package was applied to identify differentially expressed genes (DEGs). The normalization criteria include quantile normalization. DEGs were identified with adjusted *P* value < 0.05 and ∣log2 (fold change) | >1.

### 2.2. Survival Analysis

The correlation between gene expression and overall survival (OS) time was calculated using the Kaplan-Meier Plotter (http://kmplot.com/analysis/index.php?p=service&cancer=breast), which included gene expression data and survival information [14]. Results contained a hazard ratio (HR) with a 95% confidence interval (CI) and logrank *P* value.

### 2.3. Bioinformatics Analysis of DEGs

GO and KEGG analyses were conducted using the online DAVID system (https://david.ncifcrf.gov/). Significant biological processes and pathways were identified with *P* < 0.05.

### 2.4. Constructing the PPI Network

In order to explore the underlying mechanisms, we constructed PPI networks using the STRING database (http://www.string-db.org/) and visualized them using Cytoscape software.

### 2.5. Statistical Analysis

Statistical analysis was conducted using Prism V5.0 software. The *t*-test was applied. *P* < 0.05 was regarded as significant.

## 3. Results

### 3.1. Screening of DEGs in Breast Cancer

GSE26338 was used to identify DEGs in BC, which included 5 normal (NC) samples, 66 breast cancer (BC) samples, and 2 metastasis breast cancer (MBC) samples. We then conducted principal component analysis (PCA) to access the data quality of the GSE26338 database. As presented in Figure 1(a), we showed that the gene expression pattern of breast cancer and metastasis breast cancer samples was highly different from that of the normal tissues.

The genes with *P* value < 0.05 and the level that differed by ≥2-fold between two groups were defined as DEGs. As shown in Figure 1, a total of 317 DEGs were identified in this study. Cluster analysis of 317 genes identified 4 DEG clusters in breast cancer according to their expression pattern in normal samples, breast cancer samples, and metastasis breast cancer samples (Figure 1(a)). Cluster 1 included 74 DEGs, whose expression was downregulated in BC and MBC samples compared to NC samples (Figure 2(a)). Cluster 2 included 74 DEGs, whose expression was upregulated in BC and MBC samples compared to NC samples (Figure 2(b)). Cluster 3 included 91 DEGs, whose expression was downregulated in MBC compared to BC and NC samples and in BC compared to NC samples (Figure 2(c)). Cluster 4 included 78 DEGs, whose expression was overexpressed in MBC compared to BC and NC samples and in BC compared to NC samples (Figure 2(d)). These analyses suggested Cluster 1 and Cluster 2 may play a key role in the initiation of breast cancer. Cluster 3 and Cluster 4 may have a key role in both tumor initiation and metastasis of breast cancer.

### 3.2. Construction of an Integrated PPI Network

Furthermore, we constructed integrated PPI networks for Cluster 1, Cluster 2, Cluster 3, and Cluster 4 to understand the relationship among DEGs in breast cancer using the STRING database. As shown in Figure 3, we found that the Cluster 1 PPI network contained 44 nodes and 53 edges, the Cluster 2 PPI network contained 60 nodes and 281 edges, the Cluster 3 PPI network contained 19 nodes and 95 edges, and the Cluster 4 PPI network contained 20 nodes and 95 edges. ISG15, MX1, IFIT3, and SAMD9 were identified as key genes in this network, which interacted with more than 10 DEGs.

### 3.3. Function Annotation of DEGs in Cluster 3 and Cluster 4

GO analysis showed that DEGs in Cluster 3 were involved in the regulation of the molecular function, metabolic process, response to stress, cell proliferation, regulation of cell proliferation, programmed cell death, and apoptotic process (Figure 4(a)). KEGG pathway analysis showed that DEGs in Cluster 3 were related to the NOD-like receptor, Wnt, Toll-like receptor, MAPK, Neurotrophin, and Cytosolic DNA-sensing signaling (Figure 4(b)).

GO analysis showed that DEGs in Cluster 4 were involved in the viral reproductive process, mRNA metabolic process, viral reproduction, viral infectious cycle, multiorganism process, and translational initiation (Figure 4(c)). KEGG pathway analysis showed that DEGs in Cluster 4 were involved in the Toll-like receptor, RIG-I-like receptor, mRNA surveillance, Cytosolic DNA-sensing signaling, Neurotrophin, Jak-STAT, and ErbB signaling (Figure 4(d)).

### 3.4. The Abnormal Expression of Key DEGs Was Correlated to Prognosis in Breast Cancer

Furthermore, the association between the clinical outcome of patients with PCA and the expression of key DEGs was analyzed using the Kaplan-Meier Plotter. We found that higher expression of C1QB, CEP55, HIST1H2BO, IFI6, KIAA0101, PBK, SPAG5, and SPP1 and lower expression of DCN, FZD7, KRT5, and TGFBR3 were associated with shorter overall survival time in breast cancer (Figure 5).

### 3.5. Confirmation of the Abnormal Expression of Key DEGs in Breast Cancer Using TCGA Database

Then, we analyzed TCGA database to further confirm the expression levels of these hub genes in breast cancer. Our results showed that C1QB was not significantly differentially expressed in breast cancer and normal samples (Figure 6(a)). Meanwhile, we found that CEP55 (Figure 6(b)), HIST1H2BO (Figure 6(c)), IFI6 (Figure 6(d)), KIAA0101 (Figure 6(e)), PBK (Figure 6(f)), SPAG5 (Figure 6(g)), and SPP1 (Figure 6(h)) were significantly upregulated in breast cancer compared to normal samples. However, KIAA0101 (Figure 6(i)), PBK (Figure 6(j)), SPAG5 (Figure 6(k)), SPP1 (Figure 6(l)), DCN (Figure 6(m)), FZD7 (Figure 6(n)), KRT5 (Figure 6(o)), and TGFBR3 (Figure 6(p)) were scientifically downregulated in breast cancer compared to normal samples. These results were consistent with GEO dataset analysis.

### 3.6. The Upregulation of CEP55 Was Correlated to the Advanced Stage of Breast Cancer

Among these hub regulators, we focused on CEP55, which was the most significantly upregulated and was associated with the shorter overall survival time in breast cancer. In order to further confirm the clinical importance of this gene, we analyzed the correlation between CEP55 expression and clinical parameters using TCGA database. As presented in Figure 7, our analysis showed that CEP55 was remarkably upregulated in the advanced stage of breast cancer compared to the stage I breast cancer sample (Figure 7(a)). We next analyzed the expression of CEP55 in breast cancer based on subclasses. Our results showed that CEP55 was upregulated in luminal, HER2-positive, and triple-negative breast cancers compared to normal samples (Figure 7(b)). Further analysis showed that CEP55 was significantly upregulated in triple-negative breast cancers compared to other types of breast cancers, including luminal and HER2-positive cancers, demonstrating CEP55 may have a regulatory role in TNBC. Thus, we further analyzed the expression of CEP55 in different types of TNBC. Our results showed that CEP55 was the most highly expressed in Basal-like 1 TNBC and Basal-like 2 TNBC samples but the most lowly expressed in mesenchymal stem-like TNBC samples (Figure 7(c)).

## 4. Discussion

BC is the leading cause of mortality in females [1]. Distant metastasis is the main cause of BC-related death. In the past decades, there has been an urgent need to understand the mechanisms underlying BC metastasis. p38-mediated EZH2 phosphorylation could induce BC metastasis by potentiating EZH2 binding to cytoskeletal regulators [15]. OTUD1 was also identified as a metastasis-repressing factor [16]. Meanwhile, noncoding RNAs, including miRNAs and lncRNAs, were also found to play crucial roles in BC metastasis. miR-126 and miR-126^∗^ inhibited BC metastasis by recruitment of inflammatory monocytes [17]. MALAT1 acted as a BC metastasis suppressor by preventing the interaction between YAP and TEAD. lncRNA NKILA suppressed BC metastasis by blocking I*κ*B phosphorylation [18]. However, the molecular mechanisms involved in the BC spinal metastases remained largely unclear.

Recently, high-throughput methods were widely used to identify disease-related genes. Harrell et al. identified metastasis drivers involved in BC brain, lung, and liver metastases using microarray analysis. Tang et al. identified key genes involved in BC brain metastasis using GSE100534 and GSE52604. Zeng et al. identified key pathways in response to trastuzumab treatment in BC using GSE22358. Here, we conducted an analysis of the GSE26338 dataset to identify BC spinal metastasis-related key genes. A total of 317 DEGs were identified in this study. PPI networks were constructed to identify key genes. Cluster analysis showed that Cluster 3 DEGs were downregulated and Cluster 4 DEGs were upregulated in BC compared to MBC and NC samples and in MBC compared to NC samples, suggesting these DEGs play more crucial roles in BC spinal metastases. Bioinformatics analysis showed that Cluster 3 was involved in regulating the metabolic process, response to stress, cell proliferation, programmed cell death, and apoptotic process. Cluster 4 was associated with Toll-like receptor signaling and mRNA surveillance.

Of note, BC lacks effective biomarkers for screening and diagnosis. In the previous studies, a few DEGs were found to be associated with the prognosis of BC. For instance, cyclin E was found to correlate with poor disease-specific survival in BC [19]. ME1 associates with poor prognosis in BC and promotes Basal-like BC aerobic glycolysis. In order to explore the prognostic value of these DEGs, we analyzed TCGA database. We found that C1QB, CEP55, HIST1H2BO, IFI6, KIAA0101, PBK, SPAG5, and SPP1 were upregulated, while DCN, FZD7, KRT5, and TGFBR3 were suppressed in BC compared to normal samples. Kaplan-Meier curve analysis showed that higher expression of C1QB, CEP55, HIST1H2BO, IFI6, KIAA0101, PBK, SPAG5, and SPP1 and lower expression of DCN, FZD7, KRT5, and TGFBR3 were correlated to the shorter OS time in BC. In addition, we analyzed TCGA database to further confirm the expression levels of these hub genes in breast cancer. Our results showed that these regulators were significantly differentially expressed in breast cancer, which were consistent with GSE22358 dataset analysis. These findings showed that key DEGs could serve as novel biomarkers for BC.

Our above analysis identified a series of key DEGs in BC spinal metastases. Furthermore, these key DEGs were involved in regulating cancer pathways according to previous studies. C1QB was dysregulated in melanoma [20]. CEP55 was a key factor of abscission, which was found to be upregulated and correlated with the tumor stage and prognosis in multiple types of human cancers, including lung cancer [21] and colon and liver cancer [22]. IFI6 was an antiapoptosis regulator in cancer cells [23]. Previous studies showed that G1P3 (IFI6) was correlated to poor prognosis in BC, which was consistent with our finding in this study [23, 24]. Very interestingly, in breast cancer, IFI6 was revealed to promote the metastatic potential of breast cancer cells through mtROS [23]. KIAA0101 is a PCNA-associated protein, which was overexpressed in the primary lung [25], liver [26], and pancreatic carcinomas [27]. In BC, the KIAA0101 knockdown suppressed cancer cell growth by reducing cell cycle regulator expression. PBK plays a positive regulatory role in proper chromosomal separation, which is highly expressed in various types of human cancers, such as breast cancer; meanwhile, PBK was also involved in regulating the p53 and PI3K/AKT pathway. PBK had also been revealed to be a metastasis regulator in liver cancer. SPAG5 was a mitosis regulator, which interacted with Aurora-A, PLK1, and GSK3*β*. SPAG5 played crucial roles in cancer progression and was found to be upregulated in cervical, pancreatic, and lung cancers. SPP1 was a cancer metastasis regulator. In this study, we, for the first time, demonstrated that these genes were related to metastasis regulation in breast cancer, which was consistent with previous reports. Of note, multiple studies demonstrated that CEP55 had a crucial role in cancer metastasis regulation [28, 29]. For example, CEP55 promoted the migration, invasion, and neurosphere formation of the glioma cell [28], promoted epithelial-mesenchymal transition in renal cell carcinoma through the PI3K/AKT/mTOR pathway [29], and promoted migration and invasion of esophageal squamous cell carcinoma via the PI3K/AKT pathway [30]. Furthermore, our analysis demonstrated that CEP55 was remarkably upregulated in the advanced stage of breast cancer compared to the stage I breast cancer sample and was significantly upregulated in triple-negative breast cancers compared to other types of breast cancers, including luminal and HER2-positive cancers, demonstrating CEP55 may have a regulatory role in TNBC. Finally, our results showed that CEP55 was the most highly expressed in Basal-like 1 TNBC and Basal-like 2 TNBC samples but the most lowly expressed in mesenchymal stem-like TNBC samples. These reports further confirm our findings that these regulators may have an important role in cancer metastasis in breast cancer.

Also, several limitations of this study should be noted. Firstly, only 2 metastasis breast cancer (MBC) samples were included in this study. The MBC samples are limited. In future studies, more clinical MBC samples will be collected to further confirm our findings. Secondly, several key regulators were identified. However, their molecular functions remained to be unclear and need to be further confirmed using gain- or loss-of-function assays. Thirdly, the detailed mechanisms and clinical importance of CEP55 should be further explored.

## 5. Conclusion

In conclusion, this study, for the first time, screened dysregulated genes in the progression of BC spinal metastases. We also constructed PPI networks to identify key regulators in this progression. Bioinformatics analysis showed that these key regulators were involved in regulating the metabolic process, cell proliferation, Toll-like receptor pathway, and mRNA surveillance. Furthermore, our analysis revealed that key regulators were correlated to the OS time in BC patients. Although more studies are still needed to understand the functions of key regulators in BC, we provide novel information to understand the mechanisms underlying BC spinal metastases.

## Figures and Tables

**Figure 1:** Screening of differentially expressed mRNAs in BC spinal metastases. (a) PCA of GSE26338. (b) Hierarchical clustering showed differentially expressed mRNAs in the progression of BC spinal metastases.

**Figure 2:** Cluster analysis of DEGs in BC spinal metastases. (a) Cluster 1 included 87 DEGs, whose expression was downregulated in BC and MBC samples compared to NC samples. (b) Cluster 2 included 92 DEGs, whose expression was upregulated in BC and MBC samples compared to NC samples. (c) Cluster 3 included 65 DEGs, whose expression was downregulated in BC compared to MBC and NC samples and in MBC compared to NC samples. (d) Cluster 4 included 50 DEGs, whose expression was overexpressed in BC compared to MBC and NC samples and in MBC compared to NC samples.

**Figure 3:** Construction of DEG-mediated PPI networks in BC spinal metastases. (a) The Cluster 3 PPI network was identified in BC. (b) The Cluster 4 PPI network was identified in BC.

**Figure 4:** Bioinformatics analysis of DEGs in BC spinal metastases. (a, b) KEGG and GO analyses of DEGs in Cluster 3. (c, d) KEGG and GO analyses of DEGs in Cluster 4.

**Figure 5:** The dysregulation of DEGs was related to the prognosis in BC. (a–l) We observed that higher expression of C1QB, CEP55, HIST1H2BO, IFI6, KIAA0101, PBK, SPAG5, and SPP1 and lower expression of DCN, FZD7, KRT5, and TGFBR3 were correlated to shorter overall survival time in breast cancer.

**Figure 6:** Confirmation of the abnormal expression of key DEGs in breast cancer using TCGA database. (a–l) C1QB, CEP55, HIST1H2BO, IFI6, KIAA0101, PBK, SPAG5, SPP1, DCN, FZD7, KRT5, and TGFBR3 were differentially expressed in breast cancer.

**Figure 7:** The upregulation of CEP55 was correlated to the advanced stage of breast cancer. (a) CEP55 was remarkably upregulated in the advanced stage of breast cancer compared to the stage I breast cancer sample. (b) CEP55 was upregulated in luminal, HER2-positive, and triple-negative breast cancers compared to normal samples. (c) CEP55 was the most highly expressed in Basal-like 1 TNBC and Basal-like 2 TNBC samples but the most lowly expressed in mesenchymal stem-like TNBC samples.

## Data Availability

All the data analyzed in this study were downloaded from the GSE26338 dataset.
